The article "Polyurethane Elastomer Layered Nanocomposite Material for Sports Grounds and the Preparation Method Thereof" was retracted in 2023. Reasons: suspected computer-generated content; unreliable results or conclusions; concerns about the data; concerns about the results or conclusions.

# Polyurethane Elastomer Layered Nanocomposite Material for Sports Grounds and the Preparation Method Thereof

**DOI:** 10.1155/2022/5152911

**Published:** 2022-09-02

**Authors:** Chunyan Ren, Zhanguo Su, Yiping Su, Lu Wang

**Affiliations:** ^1^Faculty of Physical Education, Yulin Normal University, Yulin, 719000 Shaanxi, China; ^2^Faculty of Physical Education, Huainan Normal University, Huainan, 232038 Anhui, China; ^3^Faculty of Mathematics and Science, Universiti Pendidikan Sultan Idris, Malaysia

## Abstract

Polyurethane, as a rubber material, can relieve the load on the ground and provide seismic design for the venue, which is of great significance for sports venues. In order to improve the seismic resistance and abrasion resistance of materials for sports fields and reduce accidents in sports, this article has carried out research on the polyurethane elastomer layered nanocomposites for sports fields and their preparation. Today's world is a challenging era of science and technology. The fields of biotechnology, information, medicine, energy, environment, and national defense and security are closely related to the development of high tech, and the requirements for materials are becoming increasingly diversified. Polymer nanocomposite coating has the dual characteristics of organic and inorganic components. It not only retains the advantages of a polymer but also endows it with versatility. It meets the current application needs. It is a hot spot in today's research. Among them, there are two major problems in the composite process of nanomaterials and polymers: dispersion and compatibility. How to improve the dispersion of nanoparticles and enhance the compatibility between nanoparticles and polymers is an urgent problem to be solved. In the method part, this article introduces a small amount of polyurethane and polyurethane elastomers formed after polyurethane modification and introduces layered compounds and nanocomposites and introduces several models involved in nanomaterials in terms of algorithms. In the analysis part, this paper conducts a comprehensive analysis of the hard segment mass fraction, mechanical properties, thermal decomposition behavior, degradation mechanism, and dynamic mechanical properties. With the increase of GO content, the tensile strength increases significantly and the elongation at break becomes smaller and smaller. When the GO content increases from 0% to 2%, the tensile properties of the WPU film increase from 2.6 MPa to 7.9 MPa and the fracture of the elongation decreased from 201.7% to 62.8%. This shows that the increase in GO content will make the composite material harder and brittle. It can be seen from the experimental results that the preparation of the polyurethane elastomer layered nanocomposite material designed in this paper has a good application effect on sports venues.

The article "Polyurethane Elastomer Layered Nanocomposite Material for Sports Grounds and the Preparation Method Thereof" was retracted in 2023. Reasons: suspected computer-generated content; unreliable results or conclusions; concerns about the data; concerns about the results or conclusions.

## 1. Introduction

Nanomaterials refer to materials that have at least one dimension in the three-dimensional space at the nanometer size (1–100 nm) or are composed of them as basic units, which is approximately equivalent to the scale of 10 to 1000 atoms tightly packed together. Nanomaterials will be one of the increasingly popular materials. In recent years, the development of nanomaterials and nanostructures has made obvious achievements in the scientific research community. Nanomaterials have been successfully promoted to the most dynamic research content in the field of new material research and development and have a significant impact on the development of the society. The innovative research of new materials is the most influential strategic research field in the coming decades or even centuries, and it is of great significance to the revitalization of the economy, the development of the society, and the enhancement of national power. Biotechnology, information, medicine, energy, environment, national defense, national security, and high-tech development are inseparable, and material needs are increasingly diversified. Due to the miniaturization, advanced integration, intelligence collection, ultrafast transmission speed, and high storage density of digital information components, the material size is reduced. New military weapons, airspace, and advanced production technologies require continuous improvement in material performance. Therefore, the innovative research of new materials is the most influential strategic research field in the coming decades and even hundreds of years and is of great significance to the revitalization of the economy, the development of the society, and the enhancement of national power.

The properties of nanocomposites depend on the properties of each component, such as the shape and volume fraction of the nanofiller, the morphology of the system, and the interface interaction between the two components; the degree of performance enhancement is limited by many factors, including the aspect ratio of the nanofiller (length/diameter), its dispersion state and degree of orientation in the matrix, and the adhesiveness at the filler-matrix interface. The polyurethane's main chain structure contains repeating structural units of urethane (−NHCOO−), and it has two segments, soft segment (soft segment) and rigid segment (hard segment). PU has high strength and high elasticity. It comes from the structure of the soft and hard segments. In addition, PU also has excellent oil resistance, solvent resistance, fire resistance, and oxidation resistance. It is a polymer material widely used in industrial products. Polyurethane appeared in the 1930s. After nearly 80 years of technological development, this material has been widely used in the field of home furnishing, construction, daily necessities, transportation, and home appliances.

The article "Polyurethane Elastomer Layered Nanocomposite Material for Sports Grounds and the Preparation Method Thereof" was retracted in 2023. Reasons: suspected computer-generated content; unreliable results or conclusions; concerns about the data; concerns about the results or conclusions.

Based on the polyurethane elastomer layered nanocomposite and its preparation method, many scholars at home and abroad have conducted related research. Jiang et al. synthesized acrylate/nanozinc oxide-modified waterborne polyurethane (PUA/ZnO) to improve the wet rubbing fastness of reactive dyed cotton fabrics. The reaction conditions were optimized, and the product was characterized by FT-IR, TG, DSC, SEM, and particle size distribution. Finish the dyed cotton fabric with PUA/ZnO emulsion, and determine the rubbing fastness, UV resistance, and abrasion resistance of the treated fabric. After treatment, the wet rubbing fastness of the fabric is increased by about 0.5–1 times to 3–4 times and the ultraviolet protection factor (UPF) reaches the 50+ level. When the UPF value exceeds 50, it means that the value has reached the highest point. At this time, the knitted fabric has a good blocking effect on ultraviolet rays and the damage to the skin can be ignored. After treatment, the whiteness, air permeability, and elongation at break of the fabric did not decrease significantly. Scanning electron microscopy showed that the smooth mesh coating on the surface of the treated fabric reduced the mechanical friction between the dyed fabric and the rubbing cloth, thereby improving the rubbing fastness. The decomposition temperature of the finished fabric is increased by 50–80°C. In this study, the author conducted research on the modification of polyurethane but lacked corresponding research on various aspects of its properties such as mechanical properties [1]. Favakeh et al. synthesize dynamically crosslinked thermoplastic elastomer nanocomposites into asphalt binder-based asphalt modifiers. For linear low-density polyethylene (LLDPE) and styrene-butadiene rubber (SBR), the ratio is 80/20 and asphalt and organically modified clay (OC) are melt mixed in the presence of the sulfur vulcanization system. The suggested mixing is carried out in a closed mixer at 160 degrees Celsius with a rotor speed of 120 rpm. In order to enhance the molecular interaction between the polymer phase and the clay silicate layer, maleic anhydride grafted LLDPE (PE-g-MA) with a degree of maleation of 50% was also added to the mixture. A scanning electron microscope (SEM) was used to observe the composite samples, revealing the matrix dispersion morphology of all the dynamically vulcanized samples. X-ray diffraction (XRD) and transmission electron microscopy (TEM) examinations proved that the clay silicate layer was exfoliated and had good dispersibility. Perform rheological mechanical spectroscopy (RMS) analysis on the prepared nanocomposite material. All dynamic vulcanized nanocomposites containing 2.5% OC exhibit a shear thinning behavior and nonterminal characteristics in the low-frequency range. These indicate that the clay nanolayer forms a three-dimensional physical network in the entire LLDPE matrix. The presence of pitch in the prepared nanocomposite composition improves the fluidity of the sample. This is a promising feature of the prepared nanocomposite as an elasticity and resistance modifier in asphalt-based asphalt compositions. The author conducted related research on elastomer composite materials but did not explain the experimental characterization [2]. Under the background of comprehensive nonlinear viscoelastic contact mechanics, Abdel Rahman et al. developed a nonlinear finite element model to predict and analyze the quasistatic response of the nanoindentation problem of elastic layered viscoelastic materials with surface elastic effects. The effect of surface energy is explained by using the Gurtin-Murdoch continuum model of surface elasticity. The linear viscoelastic response is modeled by the Schapery creep model with the Prony series to express the transient component in the creep compliance. The viscoelastic constitutive equation is transformed into a recursive form, requiring only the previous time increment instead of the entire strain history. In order to accurately meet the contact constraints, the Lagrangian multiplier method is used to impose the contact conditions on the system. The balanced indentation configuration is obtained through the Newton-Raphson iterative procedure. The developed model was validated and then applied to study the quasistatic nanoindentation response of two different indentation problems with different geometries and load conditions. The results show a significant influence of surface energy and viscoelasticity on the static nanoindentation response. The author has conducted mechanical studies on the properties of elastic composite materials but has no prospects for the application of this elastic material [3].

The article "Polyurethane Elastomer Layered Nanocomposite Material for Sports Grounds and the Preparation Method Thereof" was retracted in 2023. Reasons: suspected computer-generated content; unreliable results or conclusions; concerns about the data; concerns about the results or conclusions.

The innovation of this paper lies in the preparation of polyurethane/nanosilver long-term antibacterial materials through the controlled release of Ag+. Only when nanosilver is in an aqueous environment can Ag+ be released and play an antibacterial effect. As a class of highly hydrophobic compounds, long-chain alkanes will reduce the diffusion rate of water molecules to the surface of the composite material when it is modified to the PU/Ag composite material, prolong the release time of nanosilver, and achieve a long-term antibacterial effect. Therefore, the controlled release of Ag+ can be easily achieved by adjusting the modification density of the long-chain alkyl carbene and a polyurethane-nanosilver composite material with good antibacterial properties and a long antibacterial period can be obtained. The research in this paper can provide new ideas for the preparation of layered nanopolyurethane elastomers and also provide a new direction for the related research on the improvement of nanomaterial performance.

## 2. Polyurethane Elastomer Layered Nanocomposite Material for Sports Grounds and the Preparation Method Thereof

### 2.1. Polyurethane

Polyurethane (PU) was first developed by German scientists in the 1930s. German scientists polycondensed liquid isocyanate and liquid polyether or glycol polyester to form a new type of material. Polyolefin materials are not the same; scientists named it polyurethane. Polyurethane is a block copolymer with controllable molecular weight and adjustable morphology. It has excellent comprehensive properties, such as high strength, strong load-bearing capacity, good wear resistance, excellent oil and chemical resistance, and strong load-bearing capacity under the same strength [4, 5]. Among many polymer materials, polyurethane is a material with great potential. However, with the development of production technology, various fields have put forward higher and higher requirements for materials, such as the requirements for low noise and heat preservation of EMUs. Slowly, people began to turn their attention to polyurethane/inorganic nanocomposites. For intercalated polyurethane/inorganic nanocomposites, the polymer chain is located between the clay layers, crystallization is hindered, and the conductivity of the material is improved [6]. On the other hand, the polymer is restricted by the layers, the rotation of the molecular chain and the movement of the chain segments are hindered, and the glass transition temperature of the material increases or even disappears. At the same time, the compatibility between the two phases of the inorganic sheet and the polymer is good and there is no microphase separation, so that the material exhibits special optical properties. The peeled layer is uniformly dispersed in the polymer matrix, and the compatibility between the organic-inorganic phases increases, and the mechanical strength of the material also increases [7, 8].  Figure 1 shows the schematic diagram of polyurethane.

The article "Polyurethane Elastomer Layered Nanocomposite Material for Sports Grounds and the Preparation Method Thereof" was retracted in 2023. Reasons: suspected computer-generated content; unreliable results or conclusions; concerns about the data; concerns about the results or conclusions.

### 2.2. Polyurethane Elastomer

Polyurethane elastomer (PU) is a new type of polymer material that started relatively late but developed rapidly. It took decades for polyurethane elastomers to become the forefront of the world's largest use of polymer materials. The rapid development of polyurethane elastomers is inseparable from its cheap and easy-to-obtain raw materials and simple processing and synthesis methods. Therefore, a series of polyurethane elastomers with different functions have been developed to meet the different needs of various industries for PU [9, 10]. Polyurethane elastomers are traditionally classified according to processing methods and are divided into cast polyurethane elastomers, kneading polyurethane elastomers, and thermoplastic polyurethane elastomers. At the same time, polyurethane has the characteristic that the hardness can be adjusted, so it can be obtained from hard plastic to soft elastomer products by changing different formulas. Polyurethane (PU) is one of the most important industrial materials due to its excellent tensile strength, abrasion resistance, chemical resistance, flexibility, and versatility in manufacturing. Polyurethane elastomer is composed of a hard segment and soft segment. Due to the thermodynamic incompatibility between the two phases, it is easy to separate and form a two-phase morphology in these materials. The hard segment in the polyurethane elastomer plays the role of physical crosslinking, and at the same time, it can be regarded as the high-modulus filler dispersed in the low-modulus soft segment matrix and the soft segment provides the matrix with ductility. As shown in Table 1, the hardness and tear strength of polyurethane elastomer and rubber materials are compared [11].

Polyurethane elastomer has the following characteristics:

1. The hardness control range is large. By adjusting the ratio of polyurethane raw materials or the types of raw materials, the hardness range of polyurethane can be adjusted from A0 to Shore D90 without the help of fillers. Moreover, it is commendable that high-hardness polyurethane still has good elasticity and low-hardness polyurethane also has excellent mechanical properties [12]
2. There is high mechanical strength. In the elastic interval, the ratio of tensile stress to strain is defined as the elastic modulus. Compared with other elastomers, the polyurethane elastomer has higher elastic modulus and obvious advantages. At the same time, it covers the modulus range of rubber and plastic and its tear strength is improved by more than 200% compared with rubber materials
3. Just because the polyester polyurethane elastomer has poor hydrolysis resistance than the polyether polyurethane elastomer, the hydrolysis resistance of the latter is 5 to 10 times that of the former. Under the same conditions of use, especially when water, oil, and other media exist in the working environment, the wear resistance of polyurethane elastomers is more than 10 times higher than that of other rubber materials. The protective ring in the large-scale water pump can be washed by sand for a long time without loss after being coated with polyurethane elastomer
4. There is good oil resistance. Polyurethane is highly polarized and has a weak affinity for nonpolar substances. Therefore, polyurethane elastomers are hardly corroded in the environment of nonpolar mineral oils such as kerosene, engine oil, and lubricating oil
5. There good biocompatibility. Polyurethane is a safe, nontoxic, nonhemolytic, noncoagulated, noncarcinogenic material, so it is widely used in artificial muscles, artificial blood vessels, artificial cartilage, and other artificial organs
6. There is excellent damping performance. Under the action of alternating stress, polyurethane elastomer has obvious hysteresis behavior due to energy dissipation due to molecular friction, which makes polyurethane have a good vibration and noise reduction effect. Polyurethane materials can attenuate 10%–20% of vibration energy at room temperature

The article "Polyurethane Elastomer Layered Nanocomposite Material for Sports Grounds and the Preparation Method Thereof" was retracted in 2023. Reasons: suspected computer-generated content; unreliable results or conclusions; concerns about the data; concerns about the results or conclusions.

### 2.3. Layered Compounds

Layered compounds are a class of compounds with a layered main structure, and the laminates are formed by coplanar or coedge stacking of a specific structural unit with a specific spatial structure. The layered compound is a two-dimensional plate-like structure formed by special units passing through corners, edges, and common areas. And it uses stacking vertically to create a structured three-dimensional structure. The layered structure is composed of ions or neutral molecules with different charges. The two layers of containers and plates connected by covalent bonds usually interact under the action of van der Waals forces or electrostatic properties [13, 14]. The structure model of the layered compound is shown in Figure 2.

The barrier mosaic clay in the composite material can be attributed to the volume effect and the barrier effect [15]. Laminated clay/polymer nanocomposites contain a permeable phase (amorphous polymer regions) and an impermeable phase (laminated clay and polymer crystal regions dispersed throughout the matrix). On the one hand, the polymer threshold model shows that the composite material has the same properties and performance as the pure polymer, which manifests itself as dissolved gas molecules and permeated by gas molecules. Therefore, the resolution of gas molecules decreases as the volume ratio of the substrate decreases and the layered clay effect limits the resolution of gas molecules through the composite membrane. In contrast, layered clay is impermeable to gas molecules, so layered clay can prevent the dispersion of gas molecules and extend the path of dispersion of gas molecules when they pass through the composite material. Therefore, there are three main factors that affect the relative permeability of nanocomposites: the volume fraction of layered clay, the microscopic morphology (length/width ratio), and permeability of layered clay. The number of filler particles will affect the proportion of particles per unit volume of the composite material and the number of blocking units [16, 17]. At the same time, the physical distribution of particles also plays an important role in effectively improving gas barrier properties.

The article "Polyurethane Elastomer Layered Nanocomposite Material for Sports Grounds and the Preparation Method Thereof" was retracted in 2023. Reasons: suspected computer-generated content; unreliable results or conclusions; concerns about the data; concerns about the results or conclusions.

### 2.4. Nanocomposites

When a substance keeps decreasing in size, it is below a certain critical size. The substance will acquire a series of physical and chemical properties that it does not originally possess, such as surface effects, quantum size effects, volume effects, and quantum tunneling effects [18, 19]. For most materials, this critical size is 100 nm, so the materials below the critical size are collectively called nanomaterials. There are different classification methods for nanomaterials. According to the difference in the number of dimensions in the range of 1–100 nm in the three spatial dimensions, nanomaterials are divided into three zero-dimensional materials whose dimensions are all below 100 nm, as well as corresponding one-dimensional materials and two-dimensional materials [20]. Zero-dimensional materials refer to materials in which electrons cannot move freely, such as quantum dots, nanoparticles, and powders; one-dimensional materials refer to electrons that move freely in only one nanoscale direction, such as nanowire junction materials and quantum wires. With a series of adjustable properties, users can modify nanomaterials according to their own needs, which promoted the wide application of nanomaterials in various fields such as photoelectricity, catalysis, biomedicine, analysis, and detection. Polymer nanocomposites have the following properties:

1. Mechanical properties

The mechanical properties of polymer/inorganic nanocomposites are mainly reflected in the enhancement of the material's strength, toughness, and aging resistance. Generally speaking, although polymer elastomers make the material tough, the rigidity and strength of the material are reduced and inorganic nanomaterials have the advantages of large surface area and high surface energy. Therefore, adding inorganic nanomaterials to the polymer, the mechanical properties of this composite material are stronger than those of a single polymer. The molecular chains of general polymers are easily broken under ultraviolet rays in the sun, which will cause the material to age, and some nano-oxides such as nano-SiO_2_, Al_2_O_3_, and TiO_2_ can absorb ultraviolet light of different wavelengths to reduce the material aging [21].

(2) Thermal performance

The thermal stability of polymer materials is also an important indicator for evaluating material performance. Because the thermal stability determines the performance of the polymer material against thermal degradation or aging, the single-component polymer materials have poor heat resistance and polymer-based nanocomposites can significantly improve this defect. With the addition of nanoparticles, polymerization of the thermal stability of the material-based nanocomposite is significantly improved. Nanomaterials are added to polycarbonate materials, and thermal analysis shows that the thermal stability of the composite material is significantly higher than that of a single polycarbonate material; after SiO_2_ and PC are hybridized, the thermal stability of the material is improved, and when the SiO_2_ content increases, its thermal stability also increases [22, 23].

The article "Polyurethane Elastomer Layered Nanocomposite Material for Sports Grounds and the Preparation Method Thereof" was retracted in 2023. Reasons: suspected computer-generated content; unreliable results or conclusions; concerns about the data; concerns about the results or conclusions.

In daily building construction and machine operation, the loss of materials due to vibration is very large and it is precisely because of vibration loss that the service life of materials is greatly reduced and the cost of materials is also increased. Therefore, it is very important to design a material with high shock absorption and high damping. Generally speaking, as a material for damping and vibration reduction, it is hoped that the larger the effective damping factor (the ratio of the rated load impedance of the amplifier to the actual impedance of the power amplifier), the better, and the effective damping temperature distribution range is as wide as possible, because only in this way can it be ensured that the material can be used in a certain temperature range [24, 25].

(3) Hydrophilic and hydrophobic properties

Studies have shown that adding nanocalcium carbonate to the polymer PP can increase the hydrophilicity of the polymer. At present, the main method to study the hydrophobic properties of polyurethane is to introduce chemical elements such as fluorine and silicon with hydrophobic properties into the polyurethane. The migration of electrons is restricted, and the polarizability of the CF bond is low. If there is a carbon-fluorine bond in the polymer, the intermolecular force is smaller, so the fluorine-containing polymer has a smaller surface tension and is hydrophobic. However, there are Si-O bonds with high bond energy in silicones and siloxanes are bulky and have low cohesive energy density. Therefore, silicon-containing polymers also have good hydrophobic properties [26].

The article "Polyurethane Elastomer Layered Nanocomposite Material for Sports Grounds and the Preparation Method Thereof" was retracted in 2023. Reasons: suspected computer-generated content; unreliable results or conclusions; concerns about the data; concerns about the results or conclusions.

Based on the above properties, there are also the following models for nanocomposites:

1. Nielsen model

The Nielsen model attempts to predict the macroscopic barrier based on the tortuous view [27], and the tortuous factor is defined as follows:

(1) $$\begin{array}{c} \nu =\frac{l^{\prime }}{l}=1+\frac{K}{2Z}\vartheta_{r}=1+\frac{\tau }{2}\vartheta_{r}. \end{array}$$

Among them, *l* represents the shortest distance that the penetrating molecule must traverse, *K* and *Z* represent the length and width of the layered clay, respectively, and *ϑ*_*r*_ represents the volume fraction of the layered clay in the substrate.

The influence of the tortuosity factor on permeability can be expressed as follows:

(2) $$\begin{array}{c} T_{q}=\frac{S_{\text{e}}}{S_{t}}=\frac{1-\vartheta_{r}}{\nu }, \end{array}$$

wherein it is the relative permeability and represents the permeability of the nanocomposite material and the substrate. Then, there is

(3) $$\begin{array}{c} T_{q}=\frac{\left(1-\vartheta_{r}\right)}{1+\left(\tau /2\right)\vartheta_{r}}. \end{array}$$

(2) PLN model

Assuming that each clay layer has a length of *L* and a thickness of *w*, estimate the permeability of PLN:

(4) $$\begin{array}{c} S=S_{o}\left(1-\vartheta_{r}\right)\varsigma \left(\vartheta_{r}\right). \end{array}$$

Among them, is the permeability of the substrate, andis the volume fraction of the clay layer.

Due to the restricted space environment, the movement of polymer molecular segments in PLN is obviously different from that of pure polymer, which also affects gas permeability. Therefore,

(5) $$\begin{array}{c} \varsigma \left(\vartheta_{r}\right)=\frac{\varsigma_{m}\left(\vartheta_{r}\right)}{\varsigma_{n}}. \end{array}$$

For evaluation, introducing the Nielsen model mentioned above, the tortuous path that can be traversed is as follows:

(6) $$\begin{array}{c} l^{\prime }=l_{c}+l. \end{array}$$

Among them, it represents the path that the infiltration process must traverse under the layered silicate filling, available in combination with the aforementioned model:

(7) $$\begin{array}{c} {\left(K+a\right)}^{2}\left(z+F\right)=\frac{K^{2}z}{\vartheta_{r}}. \end{array}$$

Among them, parameters *A* and *F* are the horizontal spacing and the spacing between adjacent rectangular parallelepipeds, respectively. The description path is as follows:

(8) $$\begin{array}{c} l_{c}=T_{q}\left(\frac{K}{2+{\text{l}}_{v}}\right)=\frac{l\left(K+a\right)}{2\left(z+F\right)}. \end{array}$$

The detour ratio is as follows:

(9) $$\begin{array}{c} \varsigma_{m}\left(\vartheta_{r}\right)=\frac{l}{l^{\prime }}=\frac{1}{1+{\left(1+a/K\right)}^{3}\vartheta_{r}K/2z}. \end{array}$$

The relative permeability can be expressed as follows:

(10) $$\begin{array}{c} T_{q}=\left(1-\vartheta_{r}\right)\varsigma \left(\vartheta_{r}\right)=\frac{1-\vartheta_{r}}{\varsigma_{n}\left[1+{\left(1+a/K\right)}^{3}\vartheta_{r}K/2\text{z}\right]}. \end{array}$$

It can also be expressed as follows:

(11) $$\begin{array}{c} T_{q}=\frac{\left(1-\vartheta_{r}\right)}{\varsigma_{n}\left[1+\left(K/2\right){\left(z/\vartheta_{r}\right)}^{1/2}{\left(z+F\right)}^{-3/2}\right]}. \end{array}$$

(3) Cluster model

The regular array is as follows:

(12) $$\begin{array}{c} T_{q}=\frac{\left(1-\vartheta_{r}\right)}{1+\left(1/4\right){\left(\vartheta_{r}\tau \right)}^{2}},\\ w=\overset{n}{\underset{i=1}{\sum }}R{\left(e+d\right)}^{3}\left(m+n\right)+\sqrt{b^{2}z_{r}}\varphi . \end{array}$$

The random array is as follows:

(13) $$\begin{array}{c} T_{q}=\frac{\left(1-\vartheta_{r}\right)}{1+{\left(1+\left(\vartheta_{r}\tau /3\right)\right)}^{2}},\\ u={\left(r+a\right)}^{2}\left(q+b\right)+b^{2}z_{r}. \end{array}$$

(4) Bharadwaj model

(14) $$\begin{array}{c} T_{q}=\frac{\left(1-\vartheta_{r}\right)}{1+0.667{\tau \vartheta }_{r}\left(Q+\left(1/2\right)\right)},\\ \phi =\left(1-\phi_{r}\right)\overset{n}{\underset{i=1}{\sum }}s\frac{\left(2-\phi_{r}\right)}{3+2{\tau \phi }_{r}\left(Q+\left(1/3\right)\right)}. \end{array}$$

Among them, *Q* is the orientation factor and the variation range is [−1/2, 1].

The article "Polyurethane Elastomer Layered Nanocomposite Material for Sports Grounds and the Preparation Method Thereof" was retracted in 2023. Reasons: suspected computer-generated content; unreliable results or conclusions; concerns about the data; concerns about the results or conclusions.

The static contact angle of the waterborne polyurethane nanocomposite film was measured by the JC2000CI contact angle measuring instrument. Water and ethylene glycol were used as two standard solutions to measure the surface energy of the composite film, and the material film's surface energy was calculated according to the following formula surface energy:

(15) $$\begin{array}{c} \left(1+\cos\theta \right)\gamma =4\left(\frac{\gamma_{1}^{d}\gamma_{2}^{d}}{\gamma_{2}^{d}+\gamma_{2}^{d}}+\frac{\gamma_{1}^{d}\gamma_{3}^{d}}{\gamma_{1}^{d}+\gamma_{3}^{d}}\right),\\ \left(1+\sin\theta \right)\gamma_{2}=4\left(\frac{\gamma_{3}^{d}\gamma_{2}^{d}}{\gamma_{3}^{d}+\gamma_{2}^{d}}+\frac{\gamma_{1}^{d}\gamma_{2}^{d}}{\gamma_{1}^{d}+\gamma_{2}^{d}}\right),\\ \gamma =\gamma_{1}+\gamma_{2}+\gamma_{3}. \end{array}$$

Among them, *θ*1 and *θ*2 are the contact angles of water and ethylene glycol of the material film, respectively.

## 3. Polyurethane Elastomer Layered Nanocomposite Materials for Sports Venues and Their Preparation Experiments

### 3.1. Experimental Materials and Equipment

In this paper, under the system of triethylamine, polycarbonate diol, polyether glycol, dimethylol propionic acid, and dibutyltin dilaurate, the polyurethane elastomer layered nanocomposites were prepared by the heat treatment method. The prepared materials were studied in terms of material quality, properties, thermal decomposition behavior, and degradation mechanism.

The article "Polyurethane Elastomer Layered Nanocomposite Material for Sports Grounds and the Preparation Method Thereof" was retracted in 2023. Reasons: suspected computer-generated content; unreliable results or conclusions; concerns about the data; concerns about the results or conclusions.

The experimental equipment involved in this article is shown in Table 2.

The reagents used in this article are acetylthiocholine iodide (ATChI), acetylcholinesterase (AChE), chitosan (CS deacetylation degree 85%), chloroplatinic acid (H_2_PtCl_6_·6H_2_O), FeCl_3_·6H_2_O, CH_2_Cl_2_, aniline, concentrated sulfuric acid (98%), KMnO_4_, 30% H_2_O_2_ solution, NaBH_4_, and NaNO_3_, and other drugs were purchased from the Sinopharm group. All reagents are of analytical grade. All the water used in the experiment is ultrapure water with a resistivity of 18 M*Ω*·cm. Some experimental materials are shown in Table 3.

### 3.2. Experimental Preparation Method

1. Put 7.5 g of solidified MDI and 7.9 g of polymethylene ether glycol into a 100 ml 3-neck capsule, and stir at 90° for 2 hours. Then, lower the temperature to 70°
2. Weigh 0.178 g of trimethylolpropane and 2.21 g of 1,6-hexanediol into 15 ml of acetone, and ultrasonically shake. After dissolving completely, add 0.180 g of dimethylol propionic acid to the three-necked flask, weigh 3 drops of dibutyltin dilaurate, set the temperature to 80°C, and continue the reaction for 3 hours
3. Dissolve silver nitrate solids with mass fractions of 1%, 5%, and 10% in 5 ml of DMF solvent, and shake with ultrasonic to dissolve the silver nitrate particles in DMF solvent
4. Add the dissolved silver nitrate DMF solution with different mass fractions to the polyurethane solution with a dropper, and continue to stir for 30 minutes at room temperature
5. After stirring evenly, pour it into a polytetrafluoroethylene mold and dry it with an electric dryer
6. The heat treatment process is as follows: drying at 25°C for 50 minutes ⟶ 120°C for 80 minutes ⟶ 160°C for 130 minutes ⟶ 180°C for 10 minutes

### 3.3. Characterization and Test Methods

1. The infrared spectroscopy (FTIR) instrument is as follows: EQUINOX55 Fourier Transform Infrared Spectrometer for component analysis of pure polyurethane is used. Experimental conditions are as follows: after the sample is fragile in liquid nitrogen, the absorption spectrum of the sample is measured by ATR reflection
2. The elemental analysis instrument is as follows: the elemental analyzer (VarioEL) produced by German Elementar is used to analyze the mass fraction of the hard segment in the polyurethane matrix. Experimental conditions are as follows: after the sample is dried, it is made into milligram fragments for elemental analysis
3. The particle surface morphology analysis instrument is as follows: use the NOVANanoSEM450 field emission scanning electron microscope of FEI to observe the particle morphology of the composite material
4. The composite material cross-sectional profile analysis instrument is as follows: ZEISSSUPRA55 field emission scanning electron microscope was used to observe the cross-sectional profile of composite material. Experimental conditions are as follows: after brittle fracture of the composite material sample using liquid nitrogen, the brittle fracture section was selected to prepare the observation sample. It needs to be sprayed with gold before observation, and the observation voltage is 15 kV
5. The viscoelasticity test instrument is as follows: a MCR301 rotary rheometer from Anton Paar, Austria, is used. Experimental conditions are follows: using a PP-15/E/TI/S type rotor, the test is carried out under 25°C temperature control conditions, the oscillation shear frequency is set to 1 Hz, and the strain range is set to 0.001%~100%.The stress and strain of WPU and WPU/Ag-HNT nanocomposites are shown in Table 4

The article "Polyurethane Elastomer Layered Nanocomposite Material for Sports Grounds and the Preparation Method Thereof" was retracted in 2023. Reasons: suspected computer-generated content; unreliable results or conclusions; concerns about the data; concerns about the results or conclusions.

## 4. Polyurethane Elastomer Layered Nanocomposite Materials for Sports Venues and Their Preparation Analysis

### 4.1. Hard Segment Quality Score

In this experiment, castor oil (80% to 85% ricinoleic acid, 7% oleic acid, 3% linoleic acid, 2% palmitic acid, and 1% stearic acid) is used as the soft segment raw material and diphenylmethane diisocyanate is used as the hard segment raw material. The N element only appears in the hard segment molecule, so the rigid segment in the multiblock polyurethane prepared by the experiment can be calculated by element analysis.  Table 5 is the test result table of the mass score of the polyurethane hard segment. It can be seen that the change trend of the hard segment mass score in the polyurethane sample made is in line with the experimental design trend and the actual composition of the sample is basically consistent with the design value, indicating that the experiment changed the ratio of diisocyanate and polyol in the formula. To achieve the control of the mass fraction of the rigid segment of the multiblock polyurethane, for the convenience of labeling and description, the *M* value is used to indicate the samples with different hard segment contents in the following text.

### 4.2. Mechanical Performance Analysis

Graphene oxide has a large surface area and abundant oxygen-containing groups, which can be compounded with water-based polyurethane to form a stable hydrocolloid.  Figure 3 shows the tensile stress-strain curves of WPU and GO/WPU composites. It can be seen that as the GO content increases, the tensile strength increases significantly while the elongation at break becomes smaller and smaller. When the GO content increases from 0% to 2%, the tensile properties of the WPU film increase from 2.6, the MPa increased to 7.9 MPa, and the elongation at break decreased from 201.7% to 62.8%. This shows that the increase in GO content will make the composite material harder and brittle. The reason for this phenomenon can be explained from three aspects: (i) The GO sheet is uniformly dispersed in the water-based polyurethane matrix, and the GO sheet itself has a higher specific surface area, which enhances the mechanical strength of the composite; (ii) When the GO concentration reaches a certain level, the graphene oxide sheet layer forms a relatively neat and unified self-assembled structure. Hydroxyl and epoxy groups are randomly distributed on the graphene oxide monolith, while carboxyl and carbonyl groups are introduced at the edge of the monolith. This structure can effectively enhance the tensile strength of the composite material, and the hardness will increase accordingly, resulting in the elongation at break; (iii) Reducing strong interface force between GO sheet and WPU matrix.

The article "Polyurethane Elastomer Layered Nanocomposite Material for Sports Grounds and the Preparation Method Thereof" was retracted in 2023. Reasons: suspected computer-generated content; unreliable results or conclusions; concerns about the data; concerns about the results or conclusions.

### 4.3. Thermal Decomposition Behavior Analysis

The HRR dynamic curves of pure WPU material and GO/WPU composite material are shown in Figure 4. It can be seen in Figure 4 that a large and sharp HRR peak appeared in the violent combustion of pure WPU material after being ignited and the PHRR was 573 kW/m^2^. With the increase of GO content, PHRR decreased from 573 kW/m^2^ to 527, 468, 451, and 378 kW/m^2^. When the content of GO is 2 wt%, the PHRR of the GO/WPU-2 nanocomposite is reduced by 34% compared with pure WPU material. This shows that GO has a good flame-retardant effect on the polyurethane matrix and the more content, the better the flame-retardant effect. It can also be seen that the HRR curve of WPU-1 has double peaks and WPU-2 exhibits a long flat area of the heat release curve, which indicates that GO forms a carbon layer during the combustion process, and the carbon layer acts as a good barrier. It effectively prevents heat and mass transfer.

### 4.4. Degradation Mechanism Analysis

Control the dosage of Co_3_O_4_ to 175 mg, the reaction time is 60 min, the reaction temperature is 300°C, and the content of the various products degraded by GS-MS is shown in Figure 5.

The results of GC-MS experiments showed that four degradation products, namely, p-DCB, m-DCB, o-DCB, and MCB, were obtained after the catalytic degradation of 1, 2, 4,-TrCB. In the experiment, the dissociation energy and molecular stability of the carbon-chlorine bonds in different molecules were obtained by theoretical chemistry calculations, which caused Cl(4) in 1,2,4,-TrCB to be the most difficult to remove, and Cl(2) was the easiest to remove. So, the simulation result should be: p-dichlorobenzene>m-dichlorobenzene>o-dichlorobenzene. The results obtained in this experiment are also p-dichlorobenzene>m-dichlorobenzene>o-dichlorobenzene, which just confirms the result obtained by the above theoretical calculation. Therefore, the degradation mechanism of 1, 2, 4,-TrCB in this experiment is also gradually dechlorination and hydrogenation.

The article "Polyurethane Elastomer Layered Nanocomposite Material for Sports Grounds and the Preparation Method Thereof" was retracted in 2023. Reasons: suspected computer-generated content; unreliable results or conclusions; concerns about the data; concerns about the results or conclusions.

### 4.5. Dynamic Mechanical Performance Analysis

In this experiment, nanoclay material was introduced and its dynamic mechanical properties were analyzed by analyzing the relationship between the morphology and structure of nanoclay and the structure and properties of waterborne polyurethane/clay composites.

DMA is used to analyze the relationship between the morphology and structure of nanoclay and the structure and properties of waterborne polyurethane/clay composites.  Figure 6 is a graph of the loss factor (tan*δ*) of pure WPU and WPU/clay composites. It can be seen that all samples show two tan*δ* peaks and the weaker peak at low temperature corresponds to the glass of the WPU soft segment. For transition temperature (Tgs), the stronger peak at high temperature corresponds to the glass transition temperature (Tgh) of the hard segment of WPU. The degree of microphase separation of the material can be characterized by the difference between the glass transition temperature of the hard segment and the soft segment, which is represented by ΔTg (ΔTg = Tgh − Tgs).

The data of Tgs, Tgh, and ΔTg are shown in Table 6. It can be seen that the introduction of nanoclay significantly increases the Tgs and Tgh of all samples, except for the decrease of Tgs of WPU/SHT. From the observation results of the particle surface topography analyzer, nanoclay particles are uniformly distributed in the polymer matrix. The evenly distributed nanoclay particles in the polymer matrix act as a crosslinking agent to significantly increase the crosslinking density of the composite material, and more hydrogen bonds formed in the composite material, and the strong interface formed between the modified clay, and the WPU hard segment the interaction leads to an increase in Tgh. In general, rigid inorganic nanoparticles will restrict the movement of the WPU soft segment chain and increase the Tgs of the material. However, the Tgs of WPU/SHT is lower than that of pure WPU, which may be due to the weaker interaction between SHT and WPU soft segment chains, while the stronger interaction between SHT and WPU hard segments. The study found that the ΔTg of all samples increased according to the following rule, that is, WPU < WPU/SMT < WPU/SAT < WPU/SHT. It shows that the addition of nanoclay significantly improves the degree of microphase separation of WPU/clay composites and the increase of the degree of microphase separation is consistent with the increase of ΔTg.

The article "Polyurethane Elastomer Layered Nanocomposite Material for Sports Grounds and the Preparation Method Thereof" was retracted in 2023. Reasons: suspected computer-generated content; unreliable results or conclusions; concerns about the data; concerns about the results or conclusions.

Figure 7 shows the DSC curves of different S-HBP-modified polyurethane elastomers. It can be seen that all polyurethane elastomers have a glass transition of around −40°C. It can be seen that the TMP/PU of the glass transition temperature is the highest, and the glass transition temperature moves to a low temperature with the increase of S-HBP content. At the same time, when the temperature of the curve is around 130°C, a small exothermic peak appears. This is because the isocyanate used in the synthesis of PU is diphenylmethane diisocyanate (MDI), a monomer that is easy to crystallize, so it appears at around 130°C. The exothermic peak is the crystal melting peak of the hard segment. At the same time, it can be found that as the content of S-HBP increases, the exothermic peak near 130°C in the DSC curve becomes less and less obvious. This is because the addition of S-HBP destroys the regularity of the hard segment structure, making it difficult to crystallize the hard segment that is easy to crystallize, resulting in an inconspicuous exothermic peak around 130°C. The main element content WDXRF in HNTs and Ag-HNT is shown in Table 7.

The improvement of the thermal stability of WPU composites is caused by the presence of nanomaterials. These nanoparticles act as a good thermal insulator and heat transfer barrier to make WPU composites more heat resistant.  Figure 8 shows the comparison between WPU and WPU/Ag-HNT. We can see that the thermal stability performance of the four materials is also different and the heat flow is between 14 W/g and 73 W/g, which has a significant difference.

In order to study the internal interaction between nanoparticles and composite materials, a dynamic mechanical property tester was used to test the dynamic mechanical properties of WPU and WPU/Ag-HNT nanocomposites. The comparison of energy storage effects is shown in Figure 9.

## 5. Conclusion

Polyurethane is a new material widely used in practical applications. The English name is polyurethane, which can be referred to as PU for short. It is a new type of synthetic material between plastic and rubber. It is a kind of compound containing repetitive urethane bonds in the polymer backbone. It is generally composed of polyisocyanates (mainly diisocyanates), polyols (mainly polyester polyols and polyether polyols), and small molecules. The chain agent is formed by stepwise addition polymerization. The polyurethane main chain is composed of two parts, a hard segment and a soft segment. The hard segment refers to the segment formed by the reaction of isocyanate and chain extender in the main chain of the molecule. The segment has a large volume and rigidity, while the soft segment part of it is a carbon-carbon backbone polymer polyol, which has good flexibility, and is a flexible segment in the polyurethane backbone. Changing the ratio of NCO/OH in the raw material composition ratio can adjust the molecular weight of the synthesized polyurethane and prepare polyurethane materials that can be applied to different purposes; at the same time, by changing the functionalities of isocyanates and polyols (or amines) in the polymer composition, thermoplastic polyurethane elastomers (TPUs) and thermosetting polyurethanes can be synthesized. Among them, the composition ratio of the soft segment and the hard segment in the molecular chain and its chemical structure determine the properties of the polyurethane. The microphase separation structure formed by the two makes the polyurethane have good wear resistance, fatigue resistance, and low temperature resistance. Due to the good mixing of polyurethane elastomer and nanolaminate, laminated polyurethane elastomer/nanocomposite material has good dimensional stability and barrier properties through the plane direction of nanocoating material, is a flame retardant, and will self-extinguish. When the GO content is 2 wt%, the PHRR composite of GO/WPU-2 nano is 34% less than that of pure WPU material. The special structure of this layered polymer and nanocomposite material can achieve the antibacterial effect, which is very suitable for sports venues. This paper studies and analyzes the polyurethane elastomer layered composite material used in sports fields and its preparation method and analyzes the properties of the material from multiple angles. At the same time, there are many areas that can be explored in this study, such as the absence of in-depth research on the emulsion properties of polyurethane/APU-ZnO nanocomposites, the effect of amphiphilic polyurethane-ZnO particles of different particle sizes on the antiultraviolet properties of the composite film, and applications. In the field of anti-ultraviolet, the anti-ultraviolet mechanism, anti-ultraviolet aging, and weather resistance have not been studied. In the future research work, other characteristics and application space of polyurethane materials will be continuously studied and the research quality will be continuously improved to provide more valuable research results.

The article "Polyurethane Elastomer Layered Nanocomposite Material for Sports Grounds and the Preparation Method Thereof" was retracted in 2023. Reasons: suspected computer-generated content; unreliable results or conclusions; concerns about the data; concerns about the results or conclusions.

## Figures and Tables

**Figure 1:** Schematic diagram of polyurethane.

**Figure 2:** Schematic diagram of the layered compound structure.

**Figure 3:** Tensile stress-strain curves of WPU and GO/WPU composites.

**Figure 4:** Heat release rate curves of WPU and GO/WPU nanocomposites.

**Figure 5:** Response time analysis.

**Figure 6:** Loss factor curve of WPU and WPU composite materials.

**Figure 7:** DSC curve of modified H-PU with different S-HBP contents.

**Figure 8:** Comparison between WPU and WPU/Ag-HNT.

**Figure 9:** The comparison of energy storage effects.

**Table 1:** Comparison of hardness and tear strength between polyurethane elastomer and rubber.

Performance	Polyurethane elastomer	Natural rubber	Styrene butadiene rubber
Hardness (shore A)	75–85	70–75	60–65
Tear strength	35–55	15–20	9––10

**Table 2:** Main experimental equipment used in the experiment.

Equipment name	Instrument model
Temperature programmed muffle furnace	SX2-4-10
Vacuum-drying oven	DZF-6030
Electronic balance	JA 2010
Magnetic stirrer	JA-4
Circulating water-type multipurpose vacuum pump	SHT-12C
High-speed desktop centrifuge	TGL-18D
Ultrasonic cleaner	JB-225B

**Table 3:** Part of the raw material name.

Name	Chemical formula	Specification
Triethylamine	TEA	AR
Acetone	C_3_H_6_O	AR
Polycarbonate diol	L5651-2000	Industrial products
Polyether glycol	TDIOL-1000	Industrial products
Dimethylol propionic acid	DMPA	98%
Dibutyltin dilaurate	C_32_H_64_O_4_Sn	AR

**Table 4:** The stress and strain of WPU and WPU/Ag-HNT nanocomposites.

Sample	Young's modulus (MPa)	Tensile strength (MPa)	Elongation at break (%)	Antibacterial properties (%)
WPU/Ag-HNT-0	0.9 ± 0.2	2.13 ± 0.1	4.59 ± 7.2	81.2 ± 3.7
WPU/Ag-HNT-1	2.8 ± 0.2	3.53 ± 0.1	3.56 ± 6.3	84.6 ± 3.2
WPU/Ag-HNT-2	4.6 ± 0.3	5.65 ± 0.3	2.87 ± 4.1	86.7 ± 4.7
WPU/Ag-HNT-3	12.7 ± 0.5	8.41 ± 0.3	1.82 ± 3	89.1 ± 4.1

**Table 5:** Hard segment quality score test results.

Sample serial number	1	2	3	4	5	6	7	8	9	10
Hard segment (wt%)	20.34	21.98	23.45	25.34	27.43	28.74	29.88	30.02	30.94	32.18

**Table 6:** Thermal performance and dynamic mechanical performance analysis data of WPU and WPU composite materials.

Samples	Temperature			DMA data		
	*T* (20%)	*T* (40%)	*T* (max)	TgS	Tgh	△Tg
WPU	211	357	389	-34.5	41.4	75.9
WPU/SMT	248	379	401	-23.5	59.5	83.0
WPU/SAT	229	371	399	-31.9	53.5	85.4
WPU/SHT	218	361	391	-41.8	50.6	92.4

**Table 7:** The main element content WDXRF in HNTs and Ag-HNT.

Element	Sample	
Si	Ag-HNT	HNTs
Al	29. 22	39.33
O	14.54	13.53
Fe	49.08	39.18
Ti	3.93	3.93
Ca	0.79	1.79
Mg	0.44	1.33
Ag	0.14	1.13
Others	0.105	1.115

The article "Polyurethane Elastomer Layered Nanocomposite Material for Sports Grounds and the Preparation Method Thereof" was retracted in 2023. Reasons: suspected computer-generated content; unreliable results or conclusions; concerns about the data; concerns about the results or conclusions.

## Data Availability

No data were used to support this study.
